This article has been retracted.

# Effect of 50-Hertz Sinusoidal Vibration on the Uterus in Ovariectomy-Induced Osteoporotic Rats

**DOI:** 10.1155/2022/9619867

**Published:** 2022-03-11

**Authors:** Yanfang Zhang, Yi Qi, Xianjin Zhou, FengYan Yu

**Affiliations:** ^1^Biomedical Engineering Research Laboratory, School of Information Engineering, Guangdong Medical University, Dongguan 523808, China; ^2^Guangdong Zhanjiang Institute of Marine Medicine, Zhanjiang 524023, China; ^3^The Second Clinical Medical College of Guangdong Medical University, Dongguan, Guangdong 523808, China

## Abstract

**Objective:**

To evaluate the influence of sinusoidal vibration (50-Hertz) stimulation on the uterus of osteoporotic rats.

**Methods:**

We constructed an osteoporosis rat model by ovariectomy (OVX). 36 3-month-old Sprague Dawley rats were randomly divided into the control group, vibrating group, sham operation group, sham operation vibrating group, OVX group, and OVX vibrating group (*n* = 6 per group). Rats started to vibrate one week after the operation: one 10 minutes 50-Hertz sinusoidal vibration per day, except for Saturday and Sunday. In the second, 8, and 12 week after vibration stimulation, rats were sacrificed in batches. And then, the uteruses were taken out to measure the wet weight and calculate uterus relative wet weight.

**Results:**

Compared with the control group, OVA induced a significant increase in wet weight and relative wet weight in rat uterus. The vibration was to the uterus wet weight and the uterus relative wet weight in ovariectomized rats and at the same time had no significant effect, but the 12-week prolonged vibration can significantly reduce the uterus wet weight and the uterus relative wet weight in ovariectomized rats than 2 weeks.

**Conclusions:**

The uterus wet weight and the uterus relative wet weight were increased in the OVA-induced osteoporosis rats. The 50-Hertz sinusoidal vibration had no significant effect on the uterus wet weight and the uterus relative wet weight in the ovariectomized rats at the same time, but 12 weeks of vibration can significantly reduce the uterine wet weight and uterine relative wet weight of ovariectomized rats. And the uterus relative wet weight can be used as a new indicator of stimulating the uterus.

## 1. Introduction

As the global aging population continues to increase and accelerate, it leads to an increase in chronic diseases such as osteoporosis [1]. Osteoporosis is mainly manifested by fractures, which can reduce the quality of life of patients and increase the economic burden [2]. The development of osteoporosis is associated with a variety of factors, including genetic disorders, endocrine disorders, and nutritional factors [3]. Postmenopausal estrogen deficiency is one of the causes of osteoporosis [4, 5]. In clinical practice, the common treatment for postmenopausal osteoporosis (PMOP) is hormone replacement therapy, but the increased side effects of hormone replacement therapy in patients with endometrial cancer and thrombosis make patients want to use other effective therapies with fewer side effects [6].

An integral factor in the treatment of osteoporosis should be physical therapy [7]. Vibration is a simple, economic, and effective way without drug side effects [8, 9]. Many studies have shown that vibration has obvious ability for the prevention and treatment of osteoporosis [10–12]; the ratio of P-GSK-3*β*/GSK-3*β* protein in the uterus of rats is significantly increased by treadmill and vibration, and the uterine weight index does not change significantly [13]. Kakihata et al. [14] found that mechanical vibration at 60 Hertz significantly increased bone mass in ovariectomized rats. Currently, more research is focused on the effect that vibration has on bone mineral density of ovariectomized Sprague Dawley (SD) rats [15], bone biomechanics [16], uterus [13], weight [17], and so on, but that the vibration relative to the advantages and disadvantages of drugs and other treatment of osteoporosis is less. Because vibration stimulation experiments in SD rats take a long time (up to 12 weeks), in order to reduce the impact of body weight increase on the uterus parameters during individual growth, relative wet uterus weight is introduced as a new parameter in addition to the traditional wet uterus weight parameter. Studies have shown that estrogen treatment for osteoporosis at the same time will significantly increase the uterus weight index [11, 13]. Therefore, in this study, we used 50-Hertz sinusoidal vibration for the treatment of ovariectomy- (OVX-) induced osteoporosis rats to explore the 50-Hertz sinusoidal vibration prevention and treatment of osteoporosis at the same time, whether there will be the same side effects as estrogen therapy uterine impact and to provide evidence for the prevention and treatment of osteoporosis and uterine weight changes caused by the experimental basis.

## 2. Methods and Materials

### 2.1. Animal Grouping and Surgery

This experiment selected 36 3-month-old SD female rats that had specific SPF requirement. Rats in separate cages were set at 23°C with a humidity of 80%, a clean environment, free water, and food. The standard feed that has a calcium content of 1.133% and phosphorus content of 0.195% was used. SD rats were randomly divided into 6 groups (*n* = 6 per group): control group (A), vibrating group (B), sham operation group (C), sham operation vibrating group (D), OVX group (E), and OVX vibrating group (F). The osteoporosis rat model was constructed by OVX. In brief, SD rats were placed under general anesthesia with 2% pentobarbital sodium at 0.25 ml/100 g volume to body weight ratio. Under aseptic conditions, bilateral ovaries were first removed from the rat's lateral thoracolumbar 1 cm on both sides of the longitudinal incision of the skin and muscle, and the sham operation removed ovarian volume of fat tissue. The rats were given free food and water after the operation, and according to the experiment, animals use 3R principles of humane care. This study was approved by the Animal Ethics Committee of Guangdong Medical University (GDY2012031).

### 2.2. Main Instruments and Reagents

The instrument used is the vibration table from KE BAO Test Equipment Limited Company of Dongguan, the product model is k8•F, and the manufacturing number is KB 13040219. Other instruments and reagent used were electronic scale, weighing paper, and 2% pentobarbital sodium.

### 2.3. Vibration Processing

Each day in the afternoon except Saturday and Sunday, the SD rats also began to undergo periodic sine vibration at fixed time vibration. The vibration frequency is 50 Hertz [18–20] and occurs every ten minutes. Because the SD rates began to accept the vibration one week after the operation began, the vibration of 2, 8, and 12 weeks is actually 3, 9, and 13 weeks after surgery.

### 2.4. Uterus Parameter Determination

The uterus was taken out of the SD rats and weighed in weeks 2, 8, and 12. Relatively wet uterus weight is defined as 100 ^∗^ uterus wet weight/body weight.

### 2.5. Statistical Analysis

SPSS 22.0 statistical software was used for statistical analyses. Groups were compared with a one-way ANOVA. The results were expressed as means ± standard deviation (SD). *P* values < 0.05 were considered statistically significant.

## 3. Results

### 3.1. Uterus Wet Weight

#### 3.1.1. Processing Method Comparison

In 2nd week, the uterus wet weight in group E and group F was significantly increased compared with group B and group C, and the uterus wet weight in group F was significantly increased compared with group D (*P* < 0.05). In 8th week, the uterus wet weight in group C, group E, and group F was significantly increased compared with group A, and the uterus wet weight in group F was also significantly increased compared with group B and group D. In 12th week, the uterus wet weight in group E was significantly increased compared with group A, group B, group C, and group D, and there was no statistically significant difference between the other groups (Figure 1).

#### 3.1.2. Action Time Comparison

Compared with 2nd week, the uterus wet weight in group F was significantly decreased on 12th week. With the prolongation of the duration of vibration, the uterus wet weight in groups B, D, and F decreased gradually, but there were no statistically significant differences (Figure 1).

### 3.2. The Uterus Relative Wet Weight

#### 3.2.1. Processing Method Comparison

In 2nd week, the uterus relative wet weight in group E was significantly increased compared with group B and group C, and then, the uterus relative wet weight in group F was significantly increased compared with group B, group C, and group D. In 12th week, the uterus relative wet weight in group E and group F was significantly increased compared with group A, group B, group C, and group D (Figure 2).

#### 3.2.2. Action Time Comparison

Compared with 2nd week, the uterus relative wet weight in group F was significantly decreased in 12th week, and the remaining groups had decreased but no statistically significant differences (Figure 2).

## 4. Discussion

Osteoporosis is caused by an imbalance between bone formation and bone absorption, which can not only lead to osteoporosis but also bring other diseases. As a result, older women suffer from psychosomatic disorders and a serious decline in their quality of life [21, 22]. It is known that genistein [23–26], exercise [27, 28], and whole body vibration [29–32] are several antiosteoporosis methods that have been favored by medical staff and patients in recent years. Low intensity whole body vibration training has become a new effective method for the treatment of osteoporosis [9]. Many studies [29–32] have shown that mechanical stimulation of whole body vibration is beneficial for the maintenance and increase of bone mass, confirming that vibration is indeed beneficial for the treatment of osteoporosis, but whether estrogen-like effects exist less. In this study, the model of ovariectomized rats was established. The effects of vibration and the duration of vibration on uterine wet weight and relative wet weight of uterus were observed. To understand the vibration prevention and treatment of osteoporosis at the same time, it does not produce estrogen-like effects, as well as clinical systemic vibration for the treatment of postmenopausal osteoporosis to provide more theoretical basis.

Osteoporosis causes bone mineral density, bone mass decline, and the destruction of bone microstructure by a variety of reasons, resulting in increased bone fragility, and thus prone to fracture of systemic bone disease. Osteoporosis is divided into two major categories of primary and secondary. Primary is mainly in menopausal women and the elderly as the representative of the high incidence of osteoporosis. Among them, primary osteoporosis is more harmful [9], and menopausal women and the elderly are their high-risk population. After menopause, ovarian function declines, and the secretion of estrogen will be reduced, making the role of estrogen on the promotion of endometrial and smooth muscle weakened, leading to uterine atrophy and weight loss. After menopause, ovarian function declines, further leading to the secretion of estrogen which will be reduced. It makes the promotion of estrogen on the endometrium and smooth muscle metabolism weakened, leading to uterine atrophy and weight loss.

In this experiment, six experimental groups were set up. The effects of sham operation, ovariectomization, and vibration on uterine wet weight and uterine relative wet weight in ovariectomized rats were observed at three time points of 2 weeks, 8 weeks, and 12 weeks. Compared with different treatment methods at the same time, in the initial period of vibration (2nd week), the results showed that uterine wet weight and the relative wet weight of the uterus increased significantly after ovariectomized, and vibration had no significant effect on uterine wet weight and uterine relative wet weight in ovariectomized rats; in the middle of vibration (8th week), the uterine wet weight and the relative wet weight of the uterus increased significantly after ovariectomized, and vibration had no significant effect on uterine wet weight and uterine relative wet weight in ovariectomized rats; in the late period of vibration (week 12), the uterine wet weight and the relative wet weight of the uterus increased significantly after ovariectomized, and vibration had no significant effect on uterine wet weight and uterine relative wet weight in ovariectomized rats. Compared with different treatment time at the same approach, the results showed that long-term vibration of 12 weeks could significantly reduce uterine wet weight and uterine wet weight in ovariectomized rats.

To sum up, within the same duration of vibration on uterine wet weight and uterine relative wet weight of ovariectomized rats that had no significant effect, 12 weeks of long-term vibration can make uterine wet weight and uterine relative wet weight decrease significantly. This result confirms that vibrations do not produce estrogen-like effects; that is, estrogen acts on ovariectomized rats resulting in increased uterine weight in rats [13, 33].

Vibration in the same duration of time had no significant effect on uterine wet weight and uterine relative wet weight in ovariectomized rats, which was consistent with the results of Guo et al. [13] and Hoffmann et al. [33]. But the uterine wet weight and the uterine relative wet weight increased significantly in ovariectomized rat, contrary to the research results of Guo et al. [13], Hoffmann et al. [33], and so on. The reason may be that their observation time is different after ovary, and the results need further verification. In addition, compared with the previous study, this experiment not only introduced the new parameter of relative wet weight of uterus but also investigated the effect of the different time periods on uterine wet weight and uterine relative wet weight with the same treatment factors. The results showed that long-term 12-week vibration can significantly reduce uterine wet weight and uterine relative wet weight. Exercise was beneficial to health, and ovariectomized rats lost weight after 12 weeks of uterus vibration. In the hypothetical absence of estrogen, its function can be improved and even enhanced. This corollary provides a further theoretical basis for clinical systemic vibration treatment of patients with menopausal osteoporosis, and at the same time, it triggers a brand new conjecture. Whether whole body vibration can prevent or cure other diseases, it is helpful and opens a new field to the prevention and treatment of more diseases.

## Figures and Tables

**Figure 1:** Comparison to treatment methods and effect time to OVA-induced osteoporosis rats' uterus wet weight. A, control group; B, 50-Hertz vibrating group; C, sham operation group; D, sham operation vibrating group; E, ovariectomy (OVX) group; and F, OVX vibrating group. Comparison of the treatment methods: ^∗^*P* < 0.05 and ^∗∗^*P* < 0.01 vs. group A; ^#^*P* < 0.05 and ^##^*P* < 0.01 vs. group B; ^&^*P* < 0.05 and ^&&^*P* < 0.01 vs. group C; ^^^*P* < 0.05 and ^^^^*P* < 0.01 vs. group D. Comparison of the action time: ^●^*P* < 0.05 vs. 2nd week.

**Figure 2:** Comparison to treatment methods and effect time to OVA-induced osteoporosis rats' uterus relative wet weight. A, control group; B, 50-Hertz vibrating group; C, sham operation group; D, sham operation vibrating group; E, ovariectomy (OVX) group; and F, OVX vibrating group. Comparison of the treatment methods: ^∗∗^*P* < 0.01 vs. group A; ^#^*P* < 0.05 and ^##^*P* < 0.01 vs. group B; ^&^*P* < 0.05 and ^&&^*P* <0.01 vs. group C. ^^^^*P* < 0.01 vs. group D. Comparison of the action time: ^**●**●^*P* < 0.01 vs. 2nd week.

## Data Availability

The data used to support the findings of this study are available from the corresponding author upon request.
